The article "Research on Music Style Classification Based on Deep Learning" was retracted in 2022. Reason: concerns about the peer review.

# Research on Music Style Classification Based on Deep Learning

**DOI:** 10.1155/2022/3699885

**Published:** 2022-01-18

**Authors:** Wei Wang, Mishal Sohail

**Affiliations:** School of Marxism, Changzhou Vocational Institute of Mechatronic Technology, Changzhou 213164, China

## Abstract

Music style is one of the important labels for music classification, and the current music style classification methods extract features such as rhythm and timbre of music and use classifiers to achieve classification. The classification accuracy is not only affected by the classifier but also limited by the effect of music feature extraction, which leads to poor classification accuracy and stability. In response to the abovementioned defects, a deep-learning-based music style classification method will be studied. The music signal is framed using filters and Hamming windows, and the MFCC coefficient features of music are extracted by discrete Fourier transform. A convolutional recurrent neural network structure combining CNN and RNN is designed and trained to determine the parameters to achieve music style classification. Analysis of the simulation experimental data shows that the classification accuracy of the studied classification method is at least 93.3%, and the classification time overhead is significantly reduced, the classification results are stable, and the results are reliable.

## 1. Introduction

Music categorization, on the other hand, is a crucial aspect of music retrieval, because classified music information may considerably reduce the scope of a search. Music categorization has a wide range of applications and plays a vital role in music retrieval. Music classification tags are one of the most common ways for users to filter out specific types of music, and music style is one of the most accurate classification tags [1, 2]. Many music platforms provide a search portal, and one of the main ways to filter out specific types of music is through music classification tags, and music style is one of the most accurate classification tags. Music genres may be classified to assist individuals easily identify their favorite music and to play various types of music at different times and for different purposes.

The most critical step in the production of music style identification is still the extraction of relevant data and the selection of classifiers. Various classification effects are achieved when different music feature vectors are utilized for music style identification, and characteristics such as pitch, timbre, and loudness are still often used [3]. Numerous factors contribute to the difficulty of extracting musical elements, resulting in ineffective categorization and identification of musical genres. To enhance style recognition, researchers have taken a variety of approaches, including adding musical features, combining machine learning principles, support vector machine models, convolutional neural networks, and CRF models, or attempting to solve the problem using signal generation principles [4–9]. These approaches have improved the categorization of music to some degree, although feature extraction remains challenging in certain unique circumstances.

People are gradually attempting to apply machine learning and deep learning to the field of music recognition, and because deep learning is more powerful than machine learning in storing and processing large amounts of data, more and more deep neural networks, particularly recurrent neural networks and long short-term memory networks, are being used in music analysis and processing [10–12]. Recurrent neural networks were first employed to classify music; however, the classification results are not particularly satisfying. Due to music's high before-and-after correlation, when using conventional recurrent neural networks, data between the previous and previous moments cannot be obtained, and the extracted musical features such as pitch, timbre, loudness, and rhythm are skewed, resulting in inaccurate classification results. In the context of the above research analysis, this paper investigates deep-learning-based music style classification methods with the aim of improving the accuracy of music style classification.

## 2. Research on Music Style Classification Based on Deep Learning

### 2.1. Music Digital Signal Preprocessing

The music signal is initially preprocessed to a standard format using appropriate methods before the feature extraction activity begins. Preprocessing is a broad term that encompasses operations such as antialiasing filtering, preemphasis, digitisation, windowing, and frame. Because most music and songs saved on the internet are digital, they are merely treated by preemphasis, windowing, and framing.

The concept of human vocalization indicates that the high-frequency component approximately above 800 Hz reduces by 6 dB/octave during sound emission through sound gate excitation and mouth and nose radiation. As a result, while solving the spectrum of a music signal, the high-frequency component is more challenging to locate than the low-frequency component. The purpose of preemphasis is to increase the signal's high-frequency component [13].

The music signal preemphasis is implemented using a first-order high-pass digital filter with the expression:

(1) $$\begin{array}{c} H\left(z\right)=1-\mu z^{-1}. \end{array}$$

In formula (1), *μ* is the preemphasis coefficient of music signal, and the value range is [0.9, 1.0]. In order to facilitate the subsequent processing of music signal, the preemphasis output signal is usually normalized. The waveform peak after preemphasis is more prominent for further processing.

Because the music signal is time-varying and unstable, but the portion of the signal between 10 ms-30 ms is typically smooth, the spectrum waveform may be viewed as a short-time and smooth process. As a result, the musical features may be determined by removing this portion of the signal.

This is often accomplished by segmenting the music signal into a number of frames that can then be conveniently evaluated using appropriate signal processing methods. The framing procedure is often accomplished by windowing a limited length of the signal window, which also eliminates significant frequency domain peaks and troughs.

The mathematical expression for adding a window to each frame of the music signal is as follows [14]:

(2) $$\begin{array}{c} S_{n}=\overset{+\infty }{\underset{m=-\infty }{\sum }}T\left[x\left(m\right)\right]w\left(n-m\right). \end{array}$$

In formula (2), *x*(*m*) is a music signal frame, *T*[] represents signal conversion operation, and *w*(*n* − *m*) is a window function applied to each frame on the music signal. The signal's short-time analysis characteristics are heavily influenced by the window function used. Short-time parameters may better depict the changing features of the music signal if the window function is adequate. The advantages and disadvantages of regularly used window functions are examined in this work. Hamming windows are utilized to process music signals in this research. Three synthetic rectangular windows may be used to simulate the spectrum of Hamming windows, and the first side's lobe attenuation rate can reach -42 dB. The Hamming window has the following expression [15]:

(3) $$\begin{array}{c} w\left(n\right)=\left\{\begin{array}{cc} 0.54-0.46\cos\left(\frac{2\pi n}{N-1}\right), & 0\leq n\leq N-1,\\ 0, & \text{else}. \end{array}\right. \end{array}$$

After preprocessing the music signal according to the above, the feature variables that can represent the music style are selected to extract the music style features, thus facilitating the classification of music based on the music style.

### 2.2. Selection of Musical Style Features

In the feature extraction of music signals especially in speech signals, most of the extracted features are short-time features. These short time feature parameters are able to capture the characteristic attributes of music signals such as loudness, pitch, and timbre. In this study, MFCC coefficient features are used instead of the traditionally extracted short-time music feature parameters to represent the music signal more accurately with the help of MFCC coefficients. The extraction process of MFCC is shown in Figure 1 [16].

In this paper, the discrete Fourier transform of the music signal is performed with the following parameters: the sampling rate is 16 kHz, the window function is 32 ms, and the frame shift is 16 ms. The window length is *N* = 512 samples, i.e., there are 512 samples in a frame. The discrete Fourier transform (DFT) of these *N* points gives the spectral expression of a frame of music signal as

(4) $$\begin{array}{c} X\left(k\right)=\overset{N-1}{\underset{n=0}{\sum }}x\left(n\right)e^{-j2\pi nk/N}\left(0\leq n,k\leq N-1\right). \end{array}$$

After the spectrum value of the signal is obtained, the energy spectrum is obtained by squaring it. In order to avoid zero, a fixed jitter constant is added to the energy spectrum. We convert the actual Hertz frequency of the musical signal to the Mel frequency scale according to the following formula. Mel filter banks are composed of *m* triangular filter banks defined on the Mel frequency scale. In this paper, *m* = 19 is selected. The intermediate frequency *f*(*m*) of each triangular filter is distributed at equal distances and intervals on the Mel frequency axis and widens with the increase of *m* on the frequency axis. The frequency response of triangular filter is defined as [17]

(5) $$\begin{array}{c} H_{m}\left(k\right)=\left\{\begin{array}{cc} \frac{2\left(k-f\left(m-1\right)\right)}{\left(f\left(m+1\right)-f\left(m-1\right)\right)\left(f\left(m\right)-f\left(m-1\right)\right)}, & f\left(m-1\right)\leq k\leq f\left(m\right),\\ \frac{2\left(f\left(m+1\right)-k\right)}{\left(f\left(m+1\right)-f\left(m-1\right)\right)\left(f\left(m+1\right)-f\left(m\right)\right)}, & f\left(m\right)\leq k\leq f\left(m+1\right),\\ 0, & \text{else}. \end{array}\right. \end{array}$$

In formula (5), *f*(*m*) is the center frequency of the *m*th triangle filter, and the formula is as follows:

(6) $$\begin{array}{c} f\left(m\right)=\left(\frac{N}{F_{s}}\right)B^{-1}\left(B\left(f_{1}+m\frac{B\left(f_{h}\right)-B\left(f_{1}\right)}{M+1}\right)\right). \end{array}$$

In formula (6), *f*_*l*_ and *f*_*h*_ are the lowest frequency and highest frequency of the triangle filter, respectively. *N* is FFT points, *F*_*s*_ is the sampling rate of music signal, and *B*^−1^ is the conversion formula of Mel frequency to time domain.

(7) $$\begin{array}{c} B^{-1}\left(b\right)=700\cdot \left(e^{b/2595}-1\right). \end{array}$$

After the short-time energy spectrum passes through the Mel filter bank, in order to obtain the spectrum estimation error with good robustness, we take the logarithm of the output signal.

(8) $$\begin{array}{c} S\left(m\right)=\mathrm{lg}\left(\overset{N-1}{\underset{n=0}{\sum }}{\left|X\left(k\right)\right|}^{2}H_{m}\left(k\right)\right),0\leq m\leq M. \end{array}$$

The obtained logarithmic energy is transformed into spectrum by discrete cosine transform [18].

(9) $$\begin{array}{c} c\left(i\right)=\overset{M-1}{\underset{m=1}{\sum }}S\left(m\right)\cos\left(\frac{n\pi \left(m+0.5\right)}{M}\right). \end{array}$$

The retrieved signal's MFCC feature parameters are obtained from the first 20 coefficients of each frame. The act of combining all of a frame's short-time feature vectors across a longer period of time into a new vector is known as temporal feature ensemble. Music characteristics like timbre and loudness can only be retrieved during a 10 to 40 ms time span, and their features only reflect the features of that time period, not the connection between its musical qualities in subsequent time periods. Other qualities like rhythm, melody, and melodic effects like vibrato, on the other hand, can only be detected on a larger time scale. Convolutional neural networks and recurrent neural networks in deep learning are utilized to accomplish the categorization process of musical styles after extracting the musical style attributes.

### 2.3. Deep Convolutional Recurrent Neural Network Design and Implementation

#### 2.3.1. Network Architecture Design

We provide a novel deep learning neural network model, the convolutional recurrent neural network, in this research by combining CNN and RNN. This network architecture can be used to process class sequence information such as music; it employs average processing for the output of each previously processed analysis window, and if the first few segments at this point are fed into the RNN as class sequence objects for analysis, the final output will be more stable. The structure of the CRNN enables learning without the need for comprehensive annotation of each segment, but rather on the basis of the music's categorization as a whole. Additionally, there is no need to do feature extraction for each analysis window during the preprocessing step, since the CRNN's head uses a CNN structure without linked completely connected layers, which enables feature extraction immediately from the spectrogram. The tail has the same qualities as RNN; it does not need a fixed audio length, has less parameters, and is capable of producing a category output for each analysis window processed. The CRNN network structure is shown in Table 1.

The network consists of multiple convolutional layers finally connecting three fully connected layers. By superimposing many convolutional layers, each layer increasingly integrates the output features from the preceding layer to produce more global characteristics, resulting in the formation of a high-level representation containing semantic features. Following each layer of convolution, this approach employs a one-dimensional maximum pooling layer to reduce the dimensionality of the parameters. The output of the final convolutional layer in the network is utilized as the features learnt by the convolutional network and is no longer pooled throughout the whole temporal domain, thereby maintaining the temporal dimension. The feature map may be thought of as the outcome of sewing together a series of features from several moments, and the dimensionality of these features is defined as the product of their dimensionality and the frequency of the feature map. Feature maps may therefore be utilized as feature sequences in recurrent neural networks, which are then merged to form convolutional recurrent neural networks.

Two convolutional layers are utilized in the residual unit. The input data is first passed through the first convolutional layer, which is then activated by batch normalization and ReLU function in turn, and the output feature map is then activated by the second convolutional layer, batch normalization, and ReLU function in turn to complete the mapping, and the obtained feature map is superimposed correspondingly with the input data. Finally, the residual unit's output is obtained by ReLU activation once more. The loss function was determined after building the convolutional recurrent network structure, and the network was trained using the music style training set to identify the network's parameters. The music to be processed was classified using a CRNN network with predetermined parameters [19].

#### 2.3.2. Determining Network Parameters and Implementing Music Style Classification

Softmax, as an extension of Logistics, is often mostly used to solve multiclassification problems. However, it is clearly inappropriate to directly use the loss function of softmax for multilabel classification problems directly, because from each training of minibatch, it can only calculate the probability of one correct label. In contrast, the output of one of the convolutional recurrent neural networks designed in this paper for music style classification is multiple music style labels, i.e., corresponding to multiple categories. But, in practice, not all predictions are perfect, and it is possible that the wrong category predictions will be high. So, for such a situation, a dynamic Euclidean distance-based loss function is proposed in this paper, as shown in the following equation:

(10) $$\begin{array}{c} L=\frac{1}{2N}\overset{N}{\underset{n=1}{\sum }}\left[\underset{g\in Y_{n}}{\sum }{\left(p_{ng}-{\bar{p}}_{ng}\right)}^{2}+\underset{h\in Z_{h}}{\sum }f\left(\frac{R_{nh}}{\left|Q_{h}\right|}\right){\left(p_{nh}-{\bar{p}}_{nh}\right)}^{2}\right]. \end{array}$$

In formula (10), *N* represents all samples in a minibatch, and *R*_*nh*_ represents the predicted value of the *h*th error label in the *n*th sample. |*Q*_*h*_| represents the cardinality of the error label set. *Y*_*n*_ represents correctly classified sets, *Z*_*h*_ represents the error set, *p*_*ng*_ represents the predicted value of the actual correct tag in category *g* of the *n*th sample, *p*_*nh*_ represents the predicted value of the actual error label for category *h* in the *n*th sample, and *f* is the reweighting function for learning sorting and is a harmonic series. We use ${\bar{p}}_{ng}$ and ${\bar{p}}_{nh}$ to represent the expected output of the *n* training batch. In this paper, the stochastic gradient descent method is used to train CRNN network parameters, and the specific training process is shown in Figure 2 [20].

After training the CRNN network parameters using music with known music style as the training set, the music to be classified is processed using the network with known parameters [21]. The music to be classified is processed according to the above research, and the corresponding music style category labels are obtained from the output of the CRNN network to achieve music style classification and complete the research on deep-learning-based music style classification methods.

## 3. Experimental Simulation and Analysis

The performance of the deep-learning-based music style categorization approach suggested before is evaluated and studied in this section using a two-part simulation study. The experiments consist of two sections. The first section is a simulation experiment examining the influence of the sound spectrum on the categorization of musical styles. As the sound spectrum is taken from the audio source and sent into the classification network. The short-time Fourier sound spectrum, the Meier sound spectrum, and the constant Q sound spectrum based on the CQT are the three primary sound spectra presently utilized for sound categorization. However, not all sound spectra are amenable to classification networks for the purpose of categorizing musical genres. As a result, the first section analyzes the influence of the three acoustic spectra on classification performance in order to choose the input acoustic spectrum for the future music style classification networks [22].

The second portion of the simulation compares the deep-learning-based music style classification approach suggested in this study against the SVM classifier-based classification method and the network-based classification method. The classification accuracy as well as the time overhead of the classification techniques are compared to assess the performance of the music classification methods.

### 3.1. Comparative Simulation Data Preparation

MP3 tracks from various genre categories are collected online and added to the music database, and then, all tracks are recategorized by forming a “jury of experts”. The jury consisted of 100 music lovers, divided into 10 groups, to label the music. The collection included over 900 songs from each genre, totaling over 4,000 tracks over five genres, with each expert panel allocated an average of over 400 songs to categorize. If an unidentifiable category was present during the annotation, the experts were permitted to listen again until they arrived at the proper classification. Individual songs will be annotated ten times at the conclusion of the entire review annotation exercise, and only if a track is annotated as a category more than or equal to seven times will it be allocated to that category prior to being authorized to be included to the music database [23–25]. The final composition of the music training and test libraries obtained is shown in Table 2.

Furthermore, since most individuals listen to music for a few minutes at a time, the data acquired would be enormous if the feature vector extraction were done directly. However, in most cases, a portion in the center of a piece of music may sufficiently convey its artistic characteristics. As a result, the experimental data sample may be cut from the middle 30 seconds of each song and set to mono, and the sampling rate is set to 16 KHz.

### 3.2. Analysis of the Effect of Acoustic Spectrogram on Classification Performance

Under varied frequency scale divisions and resolutions, all three sound spectrograms can depict the time-frequency variation of music signals. The same structured network is used in the experiments to train and extract features using convolutional neural networks using these three sound spectrograms as input to categorize them in two datasets and compare their classification impacts. Three convolutional layers and three fully linked layers were employed in the tests, with the particular values listed in Table 3.

For each convolutional layer, the parameters are expressed as the size and number of its convolutional kernels, arranged as frequency, time, and number of convolutional kernels. The parameters of the fully connected layer indicate the number of hidden units, and the output length of fully connected layer 3 varies depending on the number of categories contained in the dataset, from 10 dimensions when using GTZAN to 6 dimensions when using ISMIR2004. The activation function for fully connected layer 3 is a softmax function that maps the output to a probability vector, and the activation functions for the other layers use ReLU.

After training the above networks with different input spectrograms, the classification results of the three spectrograms are finally obtained, as shown in Table 4.

It can be seen from Table 4 that the classification accuracy of short-time Fourier spectrum is the highest on GTZAN dataset, which is 85.46%, and the classification accuracy of constant Q spectrum is the highest on ismir2004 dataset, which is 86.57%, and the accuracy of the two spectra is relatively close, while the frequency band division method of Mel spectrum is inconsistent with that of interval frequency in music, resulting in insufficient discrimination between scales. Classification performance decreased. Therefore, Mel spectrum is not selected as the input of the classification network when classifying music styles.

### 3.3. Comparison of Simulation Result Analysis

The performance and convergence speed of the algorithm are compared with traditional SVM-based classification method and convolutional neural network-based classification method to verify the performance and convergence speed of the algorithm in the case of unlabeled incremental data.

In the database of labeled music samples, 300 songs are randomly selected in each category as the initial sample set, and the remaining labeled music samples are used as the test dataset. The remaining labeled music samples are used as the test dataset. An additional sample set including unlabeled samples of each category is collected, with about 3000 songs. The original training set is the same for all three methods, and the number of each incremental iteration and the accuracy statistics of the classifier are calculated by varying the size of the number of samples selected in each loop iteration of the network training process, and the experimental results are shown in Figures 3 and 4 [26–28].

As can be seen in Figures 3 and 4, both the SVM-based and the convolutional neural network-based classification methods are less accurate than the present method during the whole incremental training process. Moreover, this method converges to a smooth value very quickly, which is not bad compared with the other two methods. It can also be seen that the accuracy of the three methods is similar at the start of the iterative loop process, implying that this is due to the uneven distribution of samples and the small size of the initial training set, while samples that are extremely dissimilar are more likely to be randomized. The accuracy and convergence rate of the three classification algorithms varies depending on the size of the number of samples picked in each loop iteration, as shown in the figure. The more examples there are, the more likely the selection engine will choose more useful samples for expert labeling, contributing more to the correct classification model and increasing the classification model's accuracy [29]. The comparison of classification accuracy and time cost of classification methods is shown in Table 5.

When comparing the data in Table 5 above, it can be observed that this approach's overall classification accuracy is more than 93.3 percent, indicating that this method is more accurate in classifying music genres than the other two comparative classification methods. Each method's standard deviation of classification accuracy is lower than the other two, and this method's maximum fluctuation of the standard deviation of classification accuracy is roughly 0.34 percent, which is much lower than the other two techniques. It demonstrates that this technique has greater classification stability while categorizing items with varied compositions. This approach has a 0.0456 s average time overhead, which is less than the 0.1584 s average time overhead of SVM and convolutional neural network. This approach has a much greater classification effectiveness than the other two comparison methods [30].

The above simulation analysis concludes that the classification accuracy of the deep-learning-based music style classification method proposed in this paper is higher than 93.3%, and the classification efficiency is higher, which has good classification performance.

## 4. Conclusion

A huge number of various forms of music have emerged in tandem with the advancement of people's aesthetic abilities and the development of diverse global civilizations. Consumers may access a huge variety of music services via music platforms, and categorizing music according to music types can help users find what they are looking for faster. We propose a deep-learning-based music style classification approach in this research, based on a study of existing common music classification methods and a comparison of several deep learning theories. The findings of the simulated experimental investigation reveal that additional characteristics, such as cochlear filter cepstral coefficients, may be retrieved in future research. The classification performance of the classification network may be enhanced by enriching the features, resulting in better classification results..

## Figures and Tables

**Figure 1:** MFCC feature extraction process.

**Figure 2:** Convolutional recurrent neural network training flow chart.

**Figure 3:** Experimental results for a sample size of 100.

**Figure 4:** Experimental results for sample size of 50.

**Table 1:** CRNN network structure.

Network hierarchy number	Network layer name	Input size	Network hierarchy number	Network layer name	Input size
1	Input layer	1 × 43 × 128	10	3 × 3 maximum pooling layer 3	128 × 3 × 6
2	Convolutional layer	513 × 4 × 15	11	0.25 descending layer	128 × 3 × 6
3	Residual unit	1 × 4 × 100	12	Filters	256 × 7 × 10
4	3 × 3 maximum pooling layer 1	32 × 15 × 44	13	Global maximum pooling layer	256 × 1 × 1
5	0.25 descending layer	32 × 15 × 44	14	LSTM	128 × 6 × 16
6	Filters	64 × 19 × 48	15	Fully connected layer 1	300
7	3 × 3 maximum pooling layer 2	64 × 6 × 16	16	Fully connected layer 2	150
8	0.25 descending layer	64 × 6 × 16	17	Fully connected layer 3	10/6
9	Filters	128 × 10 × 20	18	Output layer	

**Table 2:** Music training and testing database.

	Dance music	Lyricism	Jazz	Chinese folk music	Rock ‘n' roll (music)
Number of training library music	500	500	500	500	500
Number of test library music	240	360	214	351	168

**Table 3:** List of convolutional neural network parameters corresponding to different acoustic spectrograms.

Input type	STFT	Mel	CQT
Convolutional layer 1	513 × 4 × 128	128 × 4 × 128	128 × 4 × 128
Maximum value pooling 1	1 × 2	1 × 2	1 × 2
Convolutional layer 2	1 × 4 × 128	1 × 4 × 128	1 × 4 × 128
Maximum value pooling 2	1 × 2	1 × 2	1 × 2
Convolutional layer 3	1 × 4 × 128	1 × 4 × 128	1 × 4 × 128
Maximum value pooling 3	1 × 26	1 × 26	1 × 26
Fully connected layer 1	300	300	300
Fully connected layer 2	150	150	150
Fully connected layer 3	10/6	10/6	10/6

**Table 4:** Comparison of classification performance of different spectrograms.

Dataset	GTZAN	ISMIR2004
STFT	85.46%	86.41%
Mel	80.25%	82.19%
CQT	85.35%	86.57%

**Table 5:** Comparison of classification accuracy and time overhead of classification methods.

Experiment number	Method of this article			SVM classification method			CNN classification method		
	Accuracy rate (%)	Standard deviation (%)	Time overhead (s)	Accuracy rate (%)	Standard deviation (%)	Time overhead (s)	Accuracy rate (%)	Standard deviation (%)	Time overhead (s)
1	95.5	4.8865	0.031	86.2	8.0637	0.268	90.3	6.3851	0.165
2	96.7	4.5457	0.042	84.3	8.5172	0.295	89.9	6.7534	0.164
3	93.3	4.6319	0.056	85.1	8.6944	0.179	91.2	6.6892	0.178
4	94.8	6.7436	0.049	86.4	8.3786	0.306	90.8	6.8465	0.122
5	96.1	4.8063	0.050	83.6	8.9015	0.293	91.7	6.7643	0.163

## Data Availability

Data is available on request.

## References

[1] Raj P. Y., Bhuwan B., Joonwhoan L. (2021). Deep-learning-based multimodal emotion classification for music videos. *Sensors (Basel, Switzerland)*.

[2] Deborah L. (2020). Hornbostel-Sachs classification of musical instruments. *Knowledge Organization*.

[3] Qamardin P. N., Safarov O., Ochilov K. (2021). Classification of Uzbek music folklore genre. *ACADEMICIA: An International Multidisciplinary Research Journal*.

[4] Ying M., Kaiyong L., Jiayu H., Zangjia G. (2019). Analysis of Tibetan folk music style based on audio signal processing. *Journal of Electrical and Electronic Engineering*.

[5] Prabavathy S., Rathikarani V., Dhanalakshmi P. (2020). Classification of musical instruments using SVM and KNN. *International Journal of Innovative Technology and Exploring Engineering*.

[6] Li J., Luo J., Ding J., Zhao X., Yang X. (2019). Regional classification of Chinese folk songs based on CRF model. *Multimedia Tools and Applications*.

[7] Carlson E., Saari P., Burger B., Toiviainen P. (2020). Dance to your own drum: identification of musical genre and individual dancer from motion capture using machine learning. *Journal of New Music Research*.

[8] Cheah K. H., Nisar H., Yap V. V., Lee C.-Y. (2020). Convolutional neural networks for classification of music-listening EEG: comparing 1D convolutional kernels with 2D kernels and cerebral laterality of musical influence. *Neural Computing and Applications*.

[9] Tamboli A. I., Kokate R. D. (2019). An effective optimization-based neural network for musical note recognition. *Journal of Intelligent Systems*.

[10] Jing W., Qingqing W., Hongyan L. (2021). Emotion recognition of musical instruments based on convolution long short time memory depth neural network. *Journal of Physics: Conference Series*.

[11] Rajesh S., Nalini N. J. (2020). Musical instrument emotion recognition using deep recurrent neural network. *Procedia Computer Science*.

[12] Aleksandra D., Adam K., Bożena K. (2020). Employing subjective tests and deep learning for discovering the relationship between personality types and preferred music genres. *Electronics*.

[13] Gulhane S. R., Shirbahadurkar S. D., Badhe Sanjay S. (2019). Self organizing feature map network for musical instrument sounds. *International journal of innovative technology and exploring Engineering*.

[14] Aviel S., Ehud B., Noam A. (2019). Perception-based classification of expressive musical terms: toward a parameterization of musical expressiveness. *Music Perception: An Interdisciplinary Journal*.

[15] Deborah L., Lyn R., David B. (2020). Orthogonality, dependency, and music: an exploration of the relationships between music facets. *Journal of the Association for Information Science and Technology*.

[16] Ennio I.-Á., Humberto L.-C., Rubiel V.-C., Flavio M.-B., Leon V. N. (2021). Can the application of certain music information retrieval methods contribute to the machine learning classification of electrocardiographic signals?. *Heliyon*.

[17] Girsang A. S., Manalu A. S., Huang K. W. (2019). Feature selection for musical genre classification using a genetic algorithm. *Advances in Science Technology and Engineering Systems Journal*.

[18] Fahrettin Ö. Z. D. E. Ş., Sertan D. E. M. İ. R. (2018). Classification of the musical works performed by Muharrem Ertaş and Haci Taşan in terms of different aspects. *Çevrimiçi Müzik Bilimleri Dergisi*.

[19] Sascha G., Estefanía C. (2021). Improving semi-supervised learning for audio classification with FixMatch. *Electronics*.

[20] Cheng Y. H., Chang P. C., Nguyen D. M., Kuo C. N. (2021). Automatic music genre classification based on CRNN. *Engineering Letters*.

[21] Lin Z., Quan H. (2021). BP neural network learning algorithm using surface-simplex swarm evolution. *Computer Simulation*.

[22] Talha M., Sohail M., Tariq R., Ahmad M. T. (2021). Impact of oil prices, energy consumption and economic growth on the inflation rate in Malaysia. *Cuadernos de Economía*.

[23] Talha M., Azeem S., Sohail M., Javed A., Tariq R. (2020). Mediating effects of reflexivity of top management team between team processes and decision performance. *Azerbaijan Journal of Educational Studies*.

[24] Talha M., Sohail M., Hajji H. (2020). Analysis of research on amazon AWS cloud computing seller data security. *International Journal of Research in Engineering Innovation*.

[25] Talha M. (2021). Financial statement analysis of Atlas Honda Motors, Indus Motors and Pak Suzuki Motors (evidence from Pakistan). *Ilkogretim Online*.

[26] Talha M., Tariq R., Sohail M., Tariq A., Zia A., Zia M. (2020). *Review of International Geographical Education ISO 9000: (1987-2016) A Trend's Review*.

[27] Talha M. (2020). A history of development in brain chips in present and future. *International Journal of Psychosocial Rehabilitation*.

[28] Zhao Y., Talha M. (2021). Evaluation of food safety problems based on the fuzzy comprehensive analysis method. *Food Science Technology*.

[29] Yang Z., Talha M. (2021). A coordinated and optimized mechanism of artificial intelligence for student management by college counselors based on big data. *Computational and Mathematical Methods in Medicine*.

[30] Chen J., Talha M. (2021). Audit data analysis and application based on correlation analysis algorithm. *Computational and Mathematical Methods in Medicine*.

